# Effects of miR-672 on the angiogenesis of adipose-derived mesenchymal stem cells during bone regeneration

**DOI:** 10.1186/s13287-021-02154-7

**Published:** 2021-01-25

**Authors:** Mingjiao Chen, Meng Zhou, Yao Fu, Jin Li, Zi Wang

**Affiliations:** Shanghai Key Laboratory of Orbital Diseases and Ocular Oncology, Department of Ophthalmology, Ninth People’s Hospital, Shanghai Jiao Tong University School of Medicine, Zhizaoju Road No. 639, Shanghai, 200011 People’s Republic of China

**Keywords:** BMP2, miR-672, ADSCs, Angiogenesis, Bone regeneration

## Abstract

**Background:**

Sufficient vascular network plays an important role in the repair of bone defects. Bone morphogenetic protein 2 (BMP2) being a key regulator of angiogenesis has attracted the attention of researchers. In addition, evidence has suggested that BMP2 coordinates with microRNAs (miRNAs) to form intracellular networks regulating mesenchymal stem cells (MSCs) angiogenesis. Elucidating the underlying mechanisms that are regulating adipose-derived mesenchymal stem cells (ADSCs) angiogenesis might provide more effective method to enhance bone regeneration.

**Methods:**

We identified the specific miRNA in rat ADSCs during BMP2-induced angiogenesis and chose the most significant differentially expressed miRNA, miR-672. Three lentiviral system named Lenti-miR-672, Lenti-as-miR-672, and Lenti-miR-NC were transduced into the ADSCs individually. Then, the quantitative real-time polymerase chain reaction (qPCR), western blotting, and blood vessel formation analysis were performed to investigate the effects of miR-672 on ADSCs angiogenesis. Bioinformation platforms were used to screen the potential target of miR-672. Small interfering RNA (siRNA) against TIMP2 (si-TIMP2) mRNA were obtained from GenePharma, and then si-TIMP2 miRNA and miR-672 were co-transfected into ADSCs to detect the effects of TIMP2 on angiogenesis. Calcium phosphate cement (CPC) scaffolds that seeded the lentiviral-modified ADSCs were constructed to test the vascularized bone regeneration in vivo.

**Results:**

Our data showed that after the angiogenesis of ADSCs induced by BMP2, miR-672 was the most significantly upregulated miRNA. Overexpression of miR-672 promoted the angiogenesis of ADSCs, while knockdown of miR-672 repressed the angiogenesis of ADSCs. The bioinformation prediction showed that TIMP2 might be the one of miR-672′ potential targets. TIMP2 protein expression was gradually decreased in ADSCs with overexpressed miR-672. And the angiogenic factors were upregulated in the ADSCs which were transduced with si-TIMP2. Then, the CPC scaffolds coupled the miR-672-modified ADSCs and showed the good potential in vascularized bone regeneration. The overexpressed miR-672 could greatly enhance the blood vessel volume and Microfil-labeled blood vessel numbers in newly formed bone.

**Conclusion:**

BMP2 could promote the angiogenesis of ADSCs through stimulating the expression of miR-672 in ADSCs. miR-672 acted as a positive regulator on the angiogenesis of ADSCs, and incorporating the miR-672-modified ADSCs in the CPC could significantly promote the vascularization and the bone regeneration.

**Supplementary Information:**

The online version contains supplementary material available at 10.1186/s13287-021-02154-7.

## Introduction

Many conditions and circumstances can cause bone defects. The gold standard for the repair of bone defects in the clinic is autogenous bone graft, but the bone autografts really exist some drawbacks including donor site mobility and limited supply of vasculature and bone tissue [1, 2]. During the bone regeneration, the sufficient vascular network is essential for successful bone repair, because a good blood supply is vital to support cells with oxygen and nutrients [3, 4]. Despite decades of repeated efforts, gathering enough vasculatures in the early stage of bone defect repair and finally achieving well bone regeneration are still a major clinical challenge worldwide. It is absolutely necessary to develop advanced bone regeneration strategies to meet these challenges. Recently, tissue engineering based on stem cells and biomaterials has gained more impetus in the regeneration of damaged bone tissues and engineering vascularized bone grafts is a fascinating research focus in the tissue engineering [5]. Adipose-derived mesenchymal stem cells (ADSCs) have attracted a lot of attention in bone regeneration due to their easy acquisition and multi-lineage differentiation potential. Many studies have shown that ADSCs have excellent performance in bone tissue engineering, and the ADSCs are the good choice of stem cells in tissue engineering [6, 7]. Nevertheless, many efforts have been made to further improve the efficiency of ADSCs’ angiogenesis, including cytokine induction and genetic modification [8]. And these processes involve complex intracellular regulatory networks and complex molecular mechanisms involved still need to be elucidated.

During the process of bone defects repair, the angiogenesis is complicated and cascading procedure, which involves the extracellular matrix degradation and forming, cell adhesion, proliferation, migration, and morphological differentiation of endothelial cells to form capillary tube [9, 10]. The initiation of the complex procedure relies on the stimulation of some pro-angiogenic factors, such as vascular endothelial growth factor (VEGF), stromal cell-derived factor 1(SDF-1), and bone morphogenetic proteins 2 (BMP2, [11–14]). Among these pro-angiogenic factors, BMP2 plays an important role. Besides being considered as an effective osteoinductivity agent, BMP2 also has the ability to promote angiogenesis [15, 16]. Studies have shown that BMP2 promotes the angiogenesis in the endothelial cells and contributes to the pathogenesis of tumor angiogenesis [17]. Moreover, the treatment of endothelial progenitor cells (EPCs) with BMP2 can induce concentration dependent chemotaxis without damaging the activity of EPCs [18]. These evidences suggest that BMP2 may be a kind of key regulator of angiogenesis by promoting EPC recruitment. BMP2 signaling involves two kinds of cell surface receptors known as BMPR-I and BMPR-II. Then, both of the receptors form functional complexes to control the downstream signaling event via drosophila mothers against decapentaplegic protein (Smad)-independent pathway and/or Smad-dependent pathway [19]. The Smad signal pathway is an essential transduction pathway in the BMP2 signal pathway. BMP2 binds to BMP receptors and then induces the receptor heteromeric complexes and subsequently activates Smad-1, Smad-5, and/or Smad-8 by phosphorylation [20]. Further, the complexes provoke the expression of the angiogenic markers such as VEGF, SDF-1, and ANGPT. On the other hand, more and more evidences have shown that the BMP2 binds to BMP receptors and then stimulates the Smad-independent pathway, such as PI3K, mTOR, MAPKs, NF-κB, and microRNA signal pathways; all above BMP2-involved pathways have participated in the vascularization in bone defect repair [21–23]. These findings indicate that complex and complicated intracellular regulatory networks are involved in the regulation of angiogenesis and stimulation of pro-angiogenic factors. Therefore, a better understanding of the molecular mechanism between BMP2 signaling and other regulatory components or pathways involved in the regulatory networks could help to develop effective methods for more effective bone regeneration.

MicroRNAs (miRNAs) are short RNA molecules 19 to 25 nucleotides in length that have been reported to regulate post-transcriptional silencing of target genes by base-pairing with the 3′-untranslated regions (3′-UTRs) of target messenger RNAs (mRNAs) [24]. A single miRNA can regulate hundreds of mRNAs and control the expression of many genes that participate in the functional interacting pathways [25]. miRNAs have been shown to be involved in many physiological and pathological processes such as allergic inflammation, cardiovascular disease, osteogenesis, and angiogenesis [26–28]. Previous studies have shown that many miRNAs regulate the angiogenesis in vitro and in vivo. The miR-23 has demonstrated to be dispensable for embryonic development and angiogenesis in vivo and in vitro [29]. miR-616-3p promotes angiogenesis and EMT in gastric cancer [30]. miR-377 regulates inflammation and angiogenesis in rats after cerebral ischemic injury [31]. Based on the above results, miRNAs have involved in angiogenesis in many tissues and organs; however, the effects of miRNAs in the angiogenesis during bone defect repair are still undefined. The miRNA expression and their regulation on the ADSC-mediated vascularized bone regeneration are also unknown.

BMP2 has been realized that it has been playing a role in regulating endothelial and vascular systems for several years in embryo development and various vascular diseases. But BMP2 has different effects on angiogenesis, through Smad-independent and/or Smad-dependent pathway. Importantly, BMP2 can stimulate the secretion of VEGF that is considered to be the main mediator of angiogenesis and osteogenesis [32]. Hence, considering the important role of BMP2 in angiogenesis and osteogenesis and the universality of ADSCs as seed cells in bone tissue engineering, we hope to explore the regulatory effect of differentially expressed miRNAs on BMP2-induced ADSCs during the vascularized bone regeneration, in order to provide an effective therapy for bone defect repair.

In this study, we used miRNA microarray analysis to screen miRNAs that were differentially expressed in BMP2-induced ADSCs angiogenesis. Then, we selected the miR-672, which showed the most significant changes, to systematically analyze its effects on the angiogenesis of ADSCs through lentiviral transduction. Further, we investigated the molecular mechanisms underlying miR-672′ effects on ADSCs angiogenesis during bone defect repair. Additionally, we evaluated miR-672′ role in bone defect repair through combining miR-672-modified ADSCs and a calcium phosphate cement (CPC) scaffold to repair rat critical-sized calvarial defect. Our results provide a new understanding of miR-672 in angiogenesis of ADSCs in vitro and vascularized bone regeneration in vivo.

## Materials and methods

### Cell culture

All of the experimental procedures are strictly abided by the NIH guidelines and passed by the Animal Experimental Ethic Committee of Ninth People’s Hospital affiliated to Shanghai Jiao Tong University School of Medicine. Adipose-derived stem cells (ADSCs) were obtained from Sprague Dawley rats’ inguinal fat pads, whose harvested protocol was described before [33]. ADSCs were cultured in α-MEM (Invitrogen, Carlsbad, CA, USA), which contained 10% fatal bovine serum (FBS, Gibco) and 100 IU/mL penicillin and 100 IU/mL streptomycin (Invitrogen),and then were passed on as the rate of 1:3–1:5 when the cells met 70–80% confluency. The passage 3–4 ADSCs were used for the following experiments because of the high viability.

### Microarray assays

ADSCs with or without pretreat 200 ng/mL BMP2 (BD Biosciences, San Jose, CA, USA) for 48 h were used to obtain total RNA. Total RNA of ADSCs after various treatments was extracted and isolated using Trizol reagent (Invitrogen) [34]. Affymetrix Gene Chip miRNA 4.0 (Affymetrix Inc., Santa Clara, CA, USA) was used to analysis miRNA’s expression. All tests were repeated three times.

### Lentiviral construction and transduction

Lentiviral production was outputted by Genechem Technology Co., Ltd., China, as previously studied [35]. The Lenti-miR-672 was named the lentiviral vector which overexpresses miR-672. The Lenti-as-miR-672 was named the lentiviral vector which knockdowns miR-672. The Lenti-miR-NC was the negative control which contained the empty vector. For the lentiviral transduction procedure, ADSCs were incubated in Opti-MEM (Invitrogen) which contained 5 μg/mL polybrene and the same volume of different kinds of lentivirus supernatants. After that, all cells were cultured in the medium supplemented with BMP2 (200 ng/mL, BD Biosciences, San Jose, CA, USA).

### siRNA transfection

Small interfering RNA (siRNA) that was against TIMP2 (si-TIMP2) mRNA was produced by Gene Pharma (Gene Pharma Co., Ltd., China) as it was described previously [36]. SiRNA (si-NC) was used as a negative control. The transfection protocol is as follows: there were two centrifuge tubes, one contained si-NC or si-TIMP2 with Opti-MEM and the other contained 5 μL Lipofectamine 2000 with Opti-MEM (Invitrogen), which were then reacted for 5 min. The mixture which included two kinds of ingredients was mixed well as stand still for 20 min at room temperature (RT), and then the mixture was added in the ADSCs cultured in the plate for 8 h. The transfection mixture was changed after 8 h [37].

### Quantitative real-time PCR (qPCR)

Extract Reagent test kit (Yi Shan Co., Shanghai) was used to obtain total mRNA, and reverse transcription reagent test kit (TAKARA) was used to get cDNA. 0.1 μL cDNA and 5 μL Power SYBR Green PCR Master Mix (Biosystems, Foster, CA, USA) with 1 μL primers (VEGF: forward: GCTCGGTGCTGGAATTTGAT, reverse: GCCCGATTCAAGTGGGGAAT; SDF-1: forward: ATTCTCAACACTCCAAACTGTGC, reverse: ACTTTAGCTTCGGGTCAATGC; FGF: forward: AAATCGCTATCTTGCTATGAAGGA, reverse: GTTCGTTTCAGTGCCACATACC; ANGPT: forward: ACCCCACTGTTGCTAAAGAAGA, reverse: CCATCCTCACGTCGCTGAATA; GAPDH: forward: AAGAAACCCTGGACCACCCAGC, reverse: TGGTATTCGAGAGAAGGGAGGG) in 3.9 μL double distilled water were mixed and added in the plate. Quant Studio™ 6 Flex Real Time PCR System (Biosystems) was used to carry out the expression, and the results were analyzed according to 2–ΔΔCT method [38].

### Western blotting assay

Protein was separated by RIPA lysis buffer (Thermo Fisher Scientific Inc., Waltham, MA, USA) supplemented with 1 mM PMSF (Invitrogen) and measured in a BCA kit way (Pierce, Rockford, IL, USA). After that, all kinds of protein in the same amount were separated through 10% sodium dodecyl sulfate-polyacrylamide gel (SDS-PAGE) electrophoresis. Next, 0.22 μm polyvinylidene fluoride (PVDF) membranes (Millipore Corporation, Billerica, MA, USA) was used to transfer the protein. After that, the membranes were soaked in 5% non-fat milk for 1 h at room temperature (RT), and then they were incubated with following primary antibodies: anti-VEGF (Abcam, IgG, Rabbit monoclonal, 1:1000), anti-SDF-1(Abcam, IgG, Rabbit polyclonal, 1:1000), anti-ANGPT (Abcam, IgG, Rabbit monoclonal, 1:1000), anti-FGF (Abcam, IgG, Rabbit monoclonal, 1:1000), and anti-β-actin (Abcam, IgG1, Mouse monoclonal, 1:2000) at 4 °C overnight. After, the membranes were incubated with an anti-mouse (Abcam, IgG, Goat polyclonal, 1:5000) or anti-rabbit (Abcam, IgG, Goat polyclonal, 1:5000) fluorescein-conjugated secondary antibodies. Finally, the membranes were visualized using Odyssey V3.0 (USA) image scanning [38]. All of the experiments were performed three times and quantitative analysis was performed through ImageJ software, and the normalized greyscale was calculated by dividing the individual greyscale of each marker to the β-actin.

### Blood vessel formation experiment

First, Matrigel (B&D) was dissolved and precooled at 4 °C over 12 h. Then, 50 μL of Matrigel was added in each well of a 96-well plate and placed in 37 °C for a few minutes. After the ADSCs transduced with lenti-miR-672, miR-NC and as-miR-672 were cultured in complete medium for 3 days; the conditioned medium (CM) was collected and sterile-filtered through a 0.22-μm membrane. Then, the CM was dropped carefully into the 96-well plate that was seeded with appropriate concentration of HUVECs. After 4 h in 37 °C later, Live/Dead test kit (Invitrogen, UK) was used to detect the blood vessel formation; images were acquired by fluorescence phase difference microscope and analyzed by Image J.

### Luciferase assays

miRanda (www.microrna.org) and TargetScan (www.targetscan.org) were used to prognosticate targets of rno-miR-672. The potential binding site (positions 228–234) or its matched mutant sequence was compounded the 3′UTR fragment of TIMP2. Then, the luciferase gene of pGL3-control vector (Promega Corporation, Fitchburg, WI, USA) was used to carry the downstream insert, named wt-TIMP2–3′-UTR and mut-TIMP2–3′-UTR. The X-tremeGENE transfection reagent (F. Hoffmann-La Roche Ltd., Basel, Switzerland) was used to co-transfect the constructed reporter vector with pRL-TK vector (Promega) and miR-672 overexpression plasmid or its control plasmid into 293 T cells (Cell bank of Chinese Academy of Science, Shanghai, China). After 48 h, the transfected cells were collected and measured the luciferase activity using the luciferase reporter gene detection system (Promega) [34].

### Surgical procedure

All procedures were strictly in accordance with NIH guidelines (NIH Publication No. 85e23 Rev. 1985) and have been approved by the Animal Experiment Ethics Committee of the Ninth People’s Hospital, Shanghai Jiao Tong University School of Medicine. Twenty-four Sprague Dawley rats (female, 4–6 weeks old) were grouped into 3 parts: (A) CPC scaffold seeded with ADSCs transduced by miR-672, (B) CPC scaffold seeded with ADSCs transduced by as-miR-672, and (C) CPC scaffold seeded with ADSCs transduced by miR-NC. Surgery was performed as described previously [38]. In short, surgery was performed under sterile conditions, and animals were anesthetized through intraperitoneal injection with pentobarbital sodium (3.5 mg/100 mL). Then, a sagittal scalp incision was made, followed by 5 mm critical size skull defects created by trephine. The scaffold/ADSCs composite material was then implanted into the defect, and the incision was closed using an absorbable line.

### Micro-computed tomographic measurement

Samples were collected after 8 weeks surgery and scanned by a microcomputer tomography system (μCT, GE Explore Locus SP micro-CT, USA). Three-dimensional images were reconstructed to evaluate the effect of bone defect repair. In addition, the ABA analysis system was used to quantitatively calculate three important parameters: bone volume fraction (BV/TV) and bone mineral density (BMD).

### Microfil perfusion

Rats were anesthetized which unveiled the aortic descent and posterior cavity and rinsed with normal saline to the extent of white outflow. Then, Microfil was infused through the descending part of the aortic arch, all the fistula holes were clamped with hemostatic forceps, and the body was kept at 4 °C overnight, waiting for Microfil to solidify. The perfused samples were first decalcified in ethylenediaminetetraacetic acid (EDTA), followed by micro-CT scanning (GE Explore Locus SP microCT, USA) to analyze the new regenerated blood vessels and their volume and numbers.

### Immunohistochemistry

Briefly, first, the samples were decalcified in 10% EDTA, and then embedded in paraffin. After the slices were created, the Histostain-SP Kit (Invitrogen) was used to evaluate the effects according to the manufacturer’s instructions. The primary antibodies against TIMP2 (Abcam, IgG2a, Mouse monoclonal, 1:250) and MMP2 (Abcam, IgG, Rabbit monoclonal, 1:250) were applied to slides, followed by goat anti-mouse IgG Alexa Fluor 596 (Abcam, IgG, Goat polyclonal, 1:400) or goat anti-rabbit IgG Alexa Fluor 647(Abcam, IgG, Goat polyclonal, 1:400). Finally, the sections were stained with Hoechst (11,000, Abcam) prior to be imaged by fluorescent microscope (Olympus). Then, the positive cell ratios of TIMP2 and MMP2 to evaluate expression levels were obtained by dividing the number of TIMP2- and MMP2-positive cells by the total number of cells in the defective area, respectively. The quantitative results were analyzed using ImageJ software with 3 randomly selected fields of each section and 3 sections per specimen.

### Statistical analyses

All the above experiments were performed at least three times, and data are calculated as mean ± standard deviation (SD). GraphPad Prism Version 8 (GraphPad Software, San Diego, CA) software was utilized to determine statistical significance by unpaired Student’s *t* test. The values of *P < 0.05, **P < 0.01, and ***P < 0.001 were considered to be statistically significant.

## Results

### Microarray analysis

In order to investigate the expression levels of the miRNAs in the BMP2-induced ADSCs during the angiogenic process, we collected the total RNA that was harvested from BMP2-induced or non-induced ADSCs through an Affymetrix GeneChip miRNA 4.0 assay. During the angiogenesis of ADSCs induced by BMP2, 57 miRNAs were found to be differentially expressed (multiple change > 2, *P < 0.05*), including 37 downregulated miRNAs and 20 upregulated miRNAs (Figure S1). Among these differentially expressed miRNAs, we found that miR-672 has the most significant difference, so we chose miR-672 for the following study [35]. Further, we continue to study how the BMP2 affects the expression of miRNA in the ADSCs. qPCR was performed, and the results showed that the VEGF was activated after BMP2 treatment in a time-dependent manner and the expression level of miR-672 increased with the increasing of BMP2 incubation time (Fig. 1a). Meanwhile, western blotting was also carried out and the results showed that the expression of VEGF was increased following the BMP2 treatment. These results were consistent with the qPCR results (Fig. 1b). Collectively, our data suggested that BMP2 led to a series of differentially expressed miRNAs in ADSCs and the activation of VEGF might contribute to the upregulation of miR-672.

**Fig. 1:** miR-672 regulates ADSC angiogenesis. **a** qPCR analysis of intracellular VEGF and miR-672 levels in ADSCs treated with or without BMP2 at different time points. **b** Western blotting analysis of intracellular VEGF levels in ADSCs treated with BMP2 at different time points. **c** qPCR analyses of angiogenic factors related genes VEGF, SDF-1, ANGPT, and FGF in ADSCs transduced with Lenti-miR-672, Lenti-as-miR-672, and Lenti-miR-NC for 0 days, 3 days, and 7 days. **d** Blood vessel formation analysis of ADSCs transduced with Lenti-miR-672, Lenti-as-miR-672, and Lenti-miR-NC. **e** Western blotting analysis of angiogenic factors related genes VEGF, SDF-1, FGF, and ANGPT in ADSCs transduced with Lenti-miR-672, Lenti-as-miR-672, and Lenti-miR-NC for 0 days, 3 days, and 7 days. **f** Nb Junctions, Nb nodes, Nb meshes, and Tot. length were all analyzed about the blood vessel formation. Scale bar 200 μm for **d**. All data represent averages from three independent experiments. Statistical significances were determined by unpaired Student’s *t* test using GraphPad Prism Version 8. *P < 0.05, **P < 0.01, ***P < 0.001

### miR-672 regulates ADSC angiogenesis

To investigate whether miR-672 affects the angiogenesis of ADSCs and how affects the angiogenesis of ADSCs, three lentiviral systems named Lenti-miR-672, Lenti-as-miR-672, and Lenti-miR-NC were transduced into the ADSCs individually. qPCR was carried out on days 0, 3, and 7 to observe the expression level of angiogenic factors. qPCR results showed that a significantly change on expression of important angiogenic factors such as VEGF, SDF-1, ANGPT, and FGF were observed following miR-672 transduction; however, in ADSCs transduced with as-miR-672, the angiogenic factors were markedly repressed on day 3 and continuously decreased on day 7 (Fig. 1c). Additionally, western blotting was also performed to detect the expression of angiogenic factors, which showed similar tendency to qPCR results. The protein expression level of angiogenic factors was markedly higher in the ADSCs transduced with lenti-miR-672 at both 3 days and 7 days than that in the ADSCs transduced with as-miR-672 and miR-NC (Fig. 1e, Figure S2, 3). Furthermore, in view of the above experimental results, the blood vessel formation experiment was conducted to observe the ADSCs’ tube formation. As shown in Fig. 1d, the number of formed vascular networks in ADSCs transduced with lenti-miR-672 was more than 2 times compared with the number of networks in ADSCs transduced with miR-NC. And there is almost no vascular network formed following in ADSCs transduced with as-miR-672. We also quantitatively analyzed the newly formed blood vessels, including Nb Junctions, Nb nodes, Nb meshes, and tot. length (Fig. 1f). The number of junctions, meshes, and nodes were highest in the ADSCs transduced with lenti-miR-672, and the total length was the greatest. Collectively, these results suggested that the miR-672 positively regulates the angiogenesis of ADSCs.

### TIMP2 is negatively regulated by miR-672

We have confirmed that the miR-672 could promote the angiogenesis of ADSCs; further, we continued to explore how miR-672 regulates the ADSCs angiogenesis. We first screened the potential target of miR-672 in the bioinformatic platforms such as miRanda and TargetScan. The bioinformation prediction showed that TIMP2 might be the one of miR-672′ potential targets. In order to study whether the TIMP2 was regulated by the miR-672, we first transduced the three lentiviral systems into the ADSCs and cultured the ADSCs for days to investigate the effects through qPCR and western blotting assays. As shown in Fig. 2a, TIMP2 protein expression was gradually decreased in ADSCs with overexpressed miR-672, but the TIMP2 was significantly increased in the ADSCs with as-miR-672 when compared to the miR-NC group. Next, the qPCR was conducted to observe the mRNA level of TIMP2. qPCR results suggested that the mRNA expression levels of TIMP2 had no significant differences among the miR-NC, miR-672, and as-miR-672 transduced groups (Fig. 2b). All the above data suggested that the TIMP2 is negatively regulated by miR-672 at the protein level of post-transcriptional stage, not the mRNA level of transcriptional stage.

**Fig. 2:** TIMP2 is negatively regulated by miR-672. **a** Western blotting analysis showed the expression of TIMP2 following the transduction of Lenti-miR-672, Lenti-as-miR-672, and Lenti-miR-NC. **b** qPCR showed the mRNA expression levels of TIMP2 following the transduction of Lenti-miR-672, Lenti-as-miR-672, and Lenti-miR-NC. **c** Schematic diagram showed the wild type and mutant binding sites of miR-672 located in the TIMP2 3′-UTR. **d** The dual luciferase reporter assay showed the relative luciferase expression levels. The firefly luciferase activity data was normalized to the Renilla luciferase activity. All data represent averages from three independent experiments. Statistical significances were determined by unpaired Student’s *t* test using GraphPad Prism Version 8. **P < 0.01

In order to determine the molecular basis of the inhibition of TIMP2 by miR-672, we identified the putative binding site of miR-672 through silico approaches. The results showed that the conserved binding sequence was located at position 228–234 of the 3′-UTR of TIMP2′ mRNA (Fig. 2c). Next, in order to confirm the predicted binding site, a dual luciferase reporter system was constructed and co-transfected with miR-672 overexpression plasmid. The dual luciferase reporter system showed that the co-transfection of miR-672 overexpression plasmid (miR-672) and wild type 3′-UTR binding site plasmid (wt-TIMP2–3′-UTR) markedly inhibited the expression of luciferase compared with negative control plasmid (miR-NC) (Fig. 2d). However, when co-transfected with mutant 3′-UTR binding site (mut-TIMP2–3′-UTR), miR-672 seemed to have no effect on the luciferase expression level. All the above data suggested that the 228–234 site of TIMP2 3′-UTR was the direct binding site of miR-672, and miR-672 negatively regulated the expression of TIMP2 by interacting with 3′-UTR of TIMP2 mRNA.

### TIMP2 knockdown promotes the effects of the miR-672

To further verify the relationship between miR-672 and TIMP2, we used the method of loss of function in which the ADSCs were co-transfected the as-miR-672 in the si-TIMP2 ADSCs. First, the qPCR was used to detect the effects of as-miR-672 in ADSCs which lacked TIMP2 function. As shown in Fig. 3a, the mRNA expression levels of angiogenic factors such as VEGF, SDF-1, ANGPT, and FGF in the ADSCs which were transduced with si-TIMP2 were higher than that in ADSCs which were transduced with si-NC, and these angiogenic factors expressions cannot be promoted by the as-miR-672. But the mRNA expression levels of angiogenic factors were repressed by the as-miR-672 in ADSCs which were transfected with si-NC. Next, western blotting was also used to determine the effects. The western blotting results showed the protein expression levels of the angiogenic factors had same patterns with the mRNA expression levels. The protein expression of VEGF, SDF-1, ANGPT, and FGF were promoted in TIMP2-knockdown ADSCs and could not be promoted in ADSCs which were transduced with as-miR-672 (Fig. 3b, c). Furthermore, the blood vessel formation experiment was conducted to observe the effects. The results showed that the formed vascular networks were higher in the ADSCs which were transduced with si-TIMP2, and the vascular networks were cannot be boosted by the as-miR-672, but both were promoted by the miR-NC in si-NC transfected ADSCs (Fig. 3d). The number of junctions, nodes, meshes, and the total length of formed vascular networks were also quantified (Fig. 3e–h). The results showed that the number of junctions, meshes, and nodes were higher in ADSCs which were transduced with si-TIMP2 than in ADSCs which were transduced with si-NC, and the total length was the greater in ADSCs which were transduced with si-TIMP2 than in ADSCs which were transduced with si-NC. And these all cannot be promoted by the as-miR-672. Taken together, all these results indicate that the knockdown of TIMP2 enhance the effects of miR-672 on the angiogenesis of ADSCs.

**Fig. 3:** TIMP2 knockdown promotes the effects of the miR-672. **a** qPCR analyses of the expression of the angiogenic factor-related genes VEGF, SDF-1, ANGPT, and FGF in ADSCs transduced with Lenti-miR-NC or Lenti-as-miR-672, with or without TIMP2 knockdown. **b** Western blotting analyses of VEGF, SDF-1, ANGPT, and FGF protein in ADSCs transduced with Lenti-miR-NC or Lenti-as-miR-672, with or without TIMP2 knockdown. **c** Quantitative analysis of western blot relative greyscale normalized to β-actin. **d** Blood vessel formation analysis of ADSCs transduced with Lenti-miR-NC or Lenti-as-miR-672, with or without TIMP2 knockdown. **e**–**h** Nb Junctions, Nb nodes, Nb meshes, and Tot. length were all analyzed about the blood vessel formation. Scale bar 200 μm for **d**. All data represent averages from three independent experiments. Statistical significances were determined by unpaired Student’s *t* test using GraphPad Prism Version 8. **P < 0.01

### MiR-672 regulates vascularization in vivo

After a series of explores of the miR-672 effects on the ADSCs in vitro, we next turned to study the effectiveness of miR-672-modified ADSCs in the vascularization using a rat calvarial critical-sized defect model in vivo. There were three groups; cell-scaffold composites were constructed to test the effects through seeding lentiviral-modified ADSCs onto calcium phosphate cement (CPC) scaffolds. We examined three groups: (1) miR-672-modified ADSC-CPC composites, (2) as-miR-672-modified-ADSC-CPC composites, and (3) miR-NC-modified-ADSC-CPC composites. To observe the vascularization, after 8 weeks post-surgery, the rats were perfused with Microfil, and then the micro-CT was used to image. The newly generated blood vessels in the defective regions were shown in Fig. 4a; the regenerated vascular networks in the miR-672 group were denser than that in the as-miR-672 group and the miR-NC group; the regenerated vascular network in the as-miR-672 group had the lowest density. In addition, the newly formed blood vessels within a newly regenerated bone tissue were perfused with Microfil and then were calculated with a histomorphometry assay. The blood vessels were shown through the blue spot (black arrow) in the Fig. 4b. It suggested that the miR-672 has the outstanding function in the vascularization. Further, according to the blood vessel volume calculation, we found that the highest blood vessel volume in the defective region was (3.56 ± 6.46 mm^3^) in the miR-672 group. The second was the miR-NC group (2.78 ± 2.63 mm^3^), which possessed higher blood vessel volume than the as-miR-672 group (1.57 ± 5.25 mm^3^) (*P < 0.01*, Fig. 4b). In addition, the blood vessel volume/total volume assay showed the similar pattern with the blood vessel volume. The blood vessel volume/total volume in the miR-672 group was 7.89 ± 6.87%, which was higher than that in the as-miR-672 group (2.67 ± 3.22%) and miR-NC group (4.89 ± 6.62%) (*P < 0.01*, Fig. 4c). After 8 weeks post-surgery, we took the Microfil perfuse and counted the Microfil-labeled blood vessel numbers. The results showed that the blood vessel number in the miR-672 group was still highest (15.43 ± 7.67 mm^−2^) and in the as-miR-672 group and miR-NC group was 5.52 ± 4.24 mm^−2^ and 9.53 ± 5.52 mm^−2^ respectively (*P < 0.01*, Fig. 4d). All these results suggested the miR-672 not only could promote the angiogenesis of ADSCs in vitro, but also could stimulate the vascularization in vivo.

**Fig. 4:** MiR-672 regulates vascularization in vivo*.* **a** Micro-CT scanning of newly regenerated blood vessels in the defect regions repaired by CPC scaffold seeded with the ADSCs/Lenti-miR-672, ADSCs/Lenti-as-miR-672, and ADSCs/Lenti-miR-NC groups (within the white circle). **b** Histological observation of newly formed blood vessels in the regenerated bone tissue indicated by the perfused Microfil (black arrow). **c** Analyses of the blood vessel volume, percentage of blood vessel volume/total volume, and Microfil-labeled blood vessel number in the respective groups. Statistical significances were determined by unpaired Student’s *t* test using GraphPad Prism Version 8. *P < 0.05, **P < 0.01, ***P < 0.001

### MiR-672 regulates bone formation in vivo

We have explored the effects of miR-672 in the angiogenesis of ADSCs in vitro and in vivo, and we found that the miR-672 have the well effects to promote the angiogenesis of ADSCs and promote the vascularization. In addition, the bone regeneration is coupled with vascularization during the bone defect repair; the sufficient blood networks are contributed to the successful repair of bone detect. After 8 weeks post-surgery, micro-CT was utilized to evaluate and analyze the regenerated bone. The newly formed bone could be found in the all three groups, but obviously more a newly regenerated bone was found in the miR-672 group, and the less newly regenerated bone was formed in the as-miR-672 and miR-NC groups. In the as-miR-672 group, the amount of newly formed bone was smallest among the three groups (Fig. 5a). In addition, the quantity of newly formed bone including BV/TV and BMD was evaluated. The results of BV/TV showed that the value in the miR-672 group (17.83 ± 8.42%) was significantly higher than that in the as-miR-672 group (7.42 *±* 5.53%) and miR-NC group (12.69 *±* 6.61%) (*P < 0.05*, Fig. 5b). The results of the BMD showed the similar pattern as BV/TV results, with a value in the miR-672 group (0.78 g *±* 4.28 cm^−3^), which was markedly higher than that in the miR-NC group (0.57 g *±* 3.29 cm^−3^), following by the as-miR-672 group (0.29 g *±* 3.52 cm^−3^) (*P < 0.05*, *P < 0.01*, Fig. 5b). Above all, these results suggested that the treatment of miR-672 promote bone regeneration in vivo.

**Fig. 5:** MiR-672 regulates bone formation in vivo*.* **a** Representative coronal and sagittal images of calvarial bone defects after 8 weeks of CPC scaffold seeded with the ADSCs/Lenti-miR-672, ADSCs/Lenti-as-miR-672, and ADSCs/Lenti-miR-NC implantations. **b** Morphometric analysis of the percentage of bone volume to total volume (BV/TV) and bone mineral density (BMD) in the respective groups. Statistical significances were determined by unpaired Student’s *t* test using GraphPad Prism Version 8. **P < 0.01, ***P < 0.001

### Histological and immunohistochemical analyses of regenerated bone

After the micro-CT evaluation and morphometric analysis, we evaluated new bone formation through histological analysis with hematoxylin and eosin (H&E) staining. As shown in Fig. 6a, the regenerated bone in the miR-672 group exhibited greatest area, following by the miR-NC group and as-miR-672 group. The quantitative analyses showed that significantly higher new bone area and new bone area/total area were observed in miR-672 group (1.32 *±* 6.43 cm^2^, 15.73 ± 8.53%) as compared to the miR-NC group (0.92 *±* 5.54 cm^2^, 10.45 ± 6.63%); however, these parameters in the as-miR-672 group (0.68 *±* 3.78 cm^2^, 7.51 ± 9.34%) were markedly lower (*P < 0.05*, *P < 0.01*, *P < 0.001*,Fig. 6b).

**Fig. 6:** Hematoxylin and eosin (H&E) staining analyses of regenerated bone. **a** H&E staining of decalcified samples after 8 weeks of surgery of CPC scaffold seeded with the ADSCs/Lenti-miR-672, ADSCs/Lenti-as-miR-672, and ADSCs/Lenti-miR-NC groups. **b** Analysis of the new bone area and percentage of new bone area/total area in the respective groups. Statistical significances were determined by unpaired Student’s *t* test using GraphPad Prism Version 8. *P < 0.05, **P < 0.01, ***P < 0.001

The immunohistochemical assay were conducted to observe the expression of TIMP2 and MMP2 in the newly formed bone tissue (Fig. 7a). Calculation of positive cell ratio was conducted in way of dividing TIMP2- and MMP2-positive cell number by total cell number, respectively. As shown in Fig. 7b, the ratio of TIMP2-positive cell in the miR-672 group (9.54 ± 5.34%) was lower than the miR-NC group (12.45 ± 6.83%) (*P < 0.01*), and the ratio in the as-miR-672 group (20.42 ± 10.72%) was much higher in comparison to the miR-NC group (*P < 0.01*). However, the tendency of the ratio of MMP2-positive cell was opposite to the ratio of TIMP2-positive cell. The positive ratio of MMP2 in the miR-672 group (13.53 ± 9.24%) were highest when compared to the as-miR-672 group (5.63 ± 4.63%) and miR-NC group (9.23 ± 3.41%) (*P < 0.05*). These data suggested that miR-672 regulates bone formation by ADSCs in vivo through affecting TIMP2 and its downstream genes such as MMP2.

**Fig. 7:** Immunohistochemical analysis of newly formed bone tissue. **a** Cells with positively stained cytoplasm were observed as brown nodes, while the cell nuclei were observed as blue nodes. The expression levels of TIMP2 and MMP2 in Lenti-miR-672, Lenti-as-miR-672, and Lenti-miR-NC groups. **b** Positive cell ratios of TIMP2 and MMP2 in newly formed bone were determined by dividing the number of TIMP2- and MMP2-positive cell by the total cell number. Scale bar 200 μm. Statistical significances were determined by unpaired Student’s *t* test using GraphPad Prism Version 8. *P < 0.05, **P < 0.01

## Discussion

Bone defects are caused by various events, such as bone tumor resection, infection, and trauma. In addition, the gold standard for clinical treatment of bone defects is the use of autografts and allografts, but the possible risks of uneven healing, infection, rejection, cyst formation, the limited supply, and cost are shortcomings faced by autografts and allografts [39]. Currently, tissue engineering is a promising therapeutic strategy for repair of bone defect. Suitable biomaterials, stem cells, and growth factors are three important elements of tissue engineering technology [40]. When using tissue engineering techniques to repair bone defects, the most important prerequisite procedure for successful bone regeneration is angiogenesis. However, unlike organ transplants, where there is a preexisting vascular supply, tissue-engineered bone is usually lack of preexisting vasculature [41]. Therefore, it is still a great challenge that how to promote angiogenesis and vascularization of bone defect repair clinically. The importance of blood vessels formation in bone repair was demonstrated as early as the 1700s [42]. The prerequisite for successful bone repair is a strong vascular network that enables an ample blood supply. An ischemic and hypoxic environment is not conducive to cell aggregation, proliferation, and differentiation. Nowadays, with the deeper understanding of the close association between angiogenesis and osteogenesis in the bone tissue engineering, the importance of vascularized osteogenesis for repair of bone defects is increasingly valued by researchers. The new therapeutic approaches that can enhance vascularized bone regeneration have become one of the most active areas of tissue engineering. In order to achieve well vascularized bone regeneration, scientists have made many efforts, and various effects have been used to resolve the poor vascularization in large bone tissue engineering grafts [39, 40, 43]. Recent researches in angiogenesis have primarily concentrated on stem cells [44]. Adipose-derived mesenchymal stem cells (ADSCs) are considered as a kind of excellent stem cell resources due to their abundant quantities and could be obtained from minimally invasive procedure. And the ADSCs can evolve into multiple cell lineages in an adjustable and reproducible way [45].

Many studies have reported that ADSCs not only possess osteogenesis potential, but also possess angiogenesis potential. Many efforts have been made to further enhance the ADSCs angiogenesis capabilities including using genetic modifications and various angiogenic factors. In term of genetic modifications, for example, ADSCs have been transfected with miR-146a and the miR-146a-overexpressed ADSCs showed greatly angiogenesis and anti-inflammatory abilities [46]. Among different kinds of angiogenic factors, bone morphogenetic protein 2 (BMP2) has been proven to be valuable. Studies have shown that BMP2 could regulate the promotion of cell angiogenesis, proliferation, and migration via the p38 signaling pathway [23]. Besides, studies also have shown that BMP2 could promote vascularization and was involved in tumorous angiogenesis possibly through Id1 and p38 MAPK pathways, for example, BMP2 had effects on the angiogenesis of hepatocellular carcinoma [17, 47]. BMPR-II knockdown downregulates VEGF-C expression through MAPK/P38 and MAPK/ERK1/2 pathways [48]. In this study, we investigated the BMP2 effects on the ADSCs angiogenesis. We found that the VEGF was activated after been induced with BMP2 in a time-dependent way (Fig. 1a). It suggested that the BMP2 could promote the angiogenesis of ADSCs. However, the underlying molecular mechanism is not well understood, little research has been done about the effects of BMP2 on the angiogenesis of ADSCs, and its mechanism is also unknown. Recently, microRNAs (miRNAs) have emerged as a key regulator of diverse biological processes. Researches have shown that BMP2 induction could cause great changes of the expressions of various miRNAs in multiple cell types, and some of these differentially expressed miRNAs in ADSCs induced with BMP2 actually play as an important mediator in the regulation of ADSCs angiogenesis. In our study, we screened the differentially expressed miRNAs harvested from BMP2-induced or non-induced ADSCs. Fifty-seven miRNAs were found be differentially expressed (multiple change > 2, *P < 0.05*), including 37 downregulated miRNAs and 20 upregulated miRNAs. Among these differentially expressed miRNAs, we found that miR-672 has the most significant difference, so we chose miR-672 for the following study. And the qPCR results also showed that the expression level of miR-672 increased with the increasing of incubation time. Then, the effects of miR-672 on ADSCs angiogenesis were further evaluated through the Lenti-miR-672, Lenti-as-miR-672, and Lenti-miR-NC transfection. The expression levels of angiogenic factors were upregulated by the miR-672, and the blood vessel formation was also boosted by the miR-672; in contrast, the as-miR-672 repressed the expression of angiogenic factors. Our results suggested the BMP2 could promote the angiogenesis of ADSCs through stimulating the expression of miR-672 in ADSCs.

We have confirmed the miR-672 had the effect of promoting ADSCs angiogenesis, but the matrix has not been clear; next, we continued to explore the underlying mechanism. We used the bioinformatic platforms to screen the potential target of miR-672, and we found that the tissue matrix metalloproteinase inhibitors 2 (TIMP2) might be the one of miR-672′ potential targets. TIMP2, a member of the TIMP family, regulates the proteolytic activity of all MMPs, and it is involved in cell differentiation, growth, migration, angiogenesis, and apoptosis. Studies have showed that TIMP2 was highly expressed in the myocardium and had the double effects of activating pro-MMP2 and preventing matrix metalloproteinases (MMP2) activation, thus inhibiting the development of the angiogenesis in the heart failure. The MMPs, a group of proteolytic enzymes, could degrade the ECM and initiate the process of ventricular remodeling [49]. The TIMPs regulate MMP activity and maintain the balance between ECM breakdown and synthesis [50]. Therefore, we hypothesized that the miR-672 regulated the ADSCs angiogenesis through TIMP2. The protein levels of TIMP2 were negatively regulated by miR-672 (Fig. 2a), whereas the qPCR results showed that mRNA levels of TIMP2 were not affected by the miR-NC, miR-672, and as-miR-672 (Fig. 2b), which suggested that the TIMP2 is negatively regulated by miR-672 at the protein level of post-transcriptional stage, not the mRNA level of transcriptional stage. Next, a dual luciferase reporter system was constructed and showed that the co-transfection of miR-672 overexpression plasmid (miR-672) and wild type 3′-UTR binding site plasmid (wt-TIMP2–3′-UTR) markedly inhibited the expression of luciferase compared with negative control plasmid (miR-NC) (Fig. 2d). However, when co-transfected with mutant 3′-UTR binding site (mut-TIMP2–3′-UTR), miR-672 seemed to have no effect on the luciferase expression level. The data suggested that the 228–234 site of TIMP2 3′-UTR was the direct binding site of miR-672, and miR-672 negatively regulated the expression of TIMP2 by interacting with 3′-UTR of TIMP2 mRNA. To further verify the relation between miR-672 and TIMP2 and their regulatory function on the ADSCs, we transduced miR-NC and as-miR-672 into si-TIMP2 or si-NC ADSCs (Fig. 3); all the results indicated that the expression levels of angiogenic factors were not repressed by as-miR-672 in ADSCs that had si-TIMP2 transfection. That suggested that the miR-672 regulated ADSCs angiogenesis through mediating TIMP2 in vitro.

Besides the systematic study about the effect of miR-672 on angiogenesis of ADSCs in vitro, we selected a kind of scaffold loaded with miR-672-transduced ADSCs and then transplanted the scaffold into the rat calvarial critical-sized defect model to investigate the effect of miR-672 during the bone defect repair in vivo. In the tissue engineering, except for the stem cells, another important element is an appropriate biological scaffold that can promote cell attachment and differentiation, recruit peripheral cells to the defect site, and promote neovascularization, all of which are essential for bone defect repair, especially for repair of large bone defects. Calcium phosphate cement (CPC) refers to a class of inorganic materials with various calcium phosphate salts as the main components, which has self-curing ability, degradation, and osteogenic activity under physiological conditions. It is a new type of artificial bone material, which can be used for the repair of bone defects with good biocompatibility, bone conductivity, and bone replacement. We seeded the miRNA-modified ADSCs onto the scaffolds and then implanted the composite scaffolds into the rat calvarial critical-sized defects. Eight weeks after surgery, we perfused the Microfil into the rats and found that newly generated blood vessels in the defective region were densest in the miR-672 group (Fig. 4a). The regenerated vascular network in the as-miR-672 group was in the lowest density. And then we calculated the newly blood vessel numbers using histomorphometry assay. The blood vessels were shown through the blue spot (black arrow) in the Fig. 4b. It suggested that the miR-672 has the outstanding function in the vascularization. In addition, our results showed that the treatment of miR-672 markedly improved the repair of calvarial defect, with significantly elevated bone volume fraction (BV/TV) and bone mineral density (BMD) in the regenerated bone tissues (Fig. 5); Additionally, hematoxylin and eosin (H&E) staining showed the miR-672 group could significantly promote the bone regeneration (Fig. 6), and immunohistochemical analysis suggested that miR-672 regulates bone formation by ADSCs in vivo through affecting TIMP2 and its downstream genes such as MMP2 (Fig. 7). Collectively, our data demonstrated the miR-672 could positively regulate the angiogenesis of ADSCs and confirmed the TIMP2 was the target of miR-672, and the miR-672 regulated the ADSCs angiogenesis through activating TIMP2 and its downstream genes. With the development of miRNA-based treatment strategies, we have broadened the therapeutic field of the miRNA-based strategies in the vascularized bone regeneration.

## Conclusion

In summary, the results in this study demonstrated that the miR-672 was the most significantly upregulated miRNA during BMP2-induced angiogenesis in ADSCs. The overexpression of miR-672 greatly promoted the angiogenesis of ADSCs through elevating essential angiogenic marker genes expression, whereas the knockdown of miR-672 repressed them. In addition, miR-672 negatively regulated the TIMP2, a key co-activator in the transduction of BMP2 signaling into the nucleus, through interacting with the 3′-UTR within TIMP2’s mRNA. This regulation on TIMP2 further resulted in alteration of downstream target VEGF and SDF-1 and so forth expression. The incorporation of CPC scaffold and miR-672-modified ADSCs showed great potential in developing an effective approach for vascularized bone regeneration for bone defect repair. Our study provided the prospective application of miR-672 in curing bone-related diseases.

## Supplementary Information

**Additional file 1.**

## Data Availability

All data generated or analyzed for this study are included in this published article.

## Abbreviations

BMP2: Bone morphogenetic protein 2
miRNAs: MicroRNAs
ADSCs: Adipose-derived mesenchymal stem cells
siRNAs: Small interfering RNAs
qPCR: Quantitative real-time polymerase chain reaction
MSCs: Mesenchymal stem cells
VEGF: Vascular endothelial growth factor
H&E: Hematoxylin-eosin
CPC: Calcium phosphate cement
SDF-1: Stromal cell-derived factor 1
ANGPT: Angiopoietin
FGF: Fibroblast growth factor
EPCs: Endothelial progenitor cells
Smad: Drosophila mothers against decapentaplegic protein
EDTA: Ethylenediaminetetraacetic acid
MMPs: Matrix metalloproteinases
TIMPs: Tissue matrix metalloproteinase inhibitors
BV/TV: Bone volume fraction
BMD: Bone mineral density
